The article "Observation on Application Effect of Arterial Puncture and Catheterization under Guidance of Intelligent Medical Care Ultrasound in Clinical Anesthesia" was retracted in 2023. Reasons: signs of a paper mill; suspected computer-generated content; unreliable results or conclusions; lack of ethics approval or compliance.

# Observation on Application Effect of Arterial Puncture and Catheterization under Guidance of Intelligent Medical Care Ultrasound in Clinical Anesthesia

**DOI:** 10.1155/2022/6970274

**Published:** 2022-03-28

**Authors:** Guozhang Ren, Xiancheng Qiang, Hui Yu

**Affiliations:** ^1^Department of Anesthesiology, Yantai Hospital of Traditional Chinese Medicine, Yantai 264000, Shandong, China; ^2^Department of Anesthesiology, Qingdao Eighth Peolpe's Hospital, Qingdao 266100, Shandong, China; ^3^Department of Anesthesiology, Qingdao Eye Hospital Affiliated to Shandong First Medical Universty, Qingdao, 266071, Shandong, China

## Abstract

In clinical anesthesia and the rescue of critically ill patients, arterial puncture and catheterization are the most commonly chosen ways to establish central arterial access for patients. Invasive arterial puncture and catheterization facilitate the grasp of real-time vital sign information of patients during surgery, which strengthens patient monitoring during surgery and improves safety. However, the traditional method of arterial puncture and cannulation through palpation of the radial artery is often prone to complications related to mechanical injury, such as hemorrhage, hematoma, and accidental perforation of the artery. Studies have shown that ultrasound-guided radial artery puncture and cannulation can shorten the puncture cannulation time, reduce the incidence of complications related to puncture cannulation, and improve the success rate of puncture cannulation. In order to verify it, this paper uses the experimental group and the control group to conduct comparative experiments and uses the neural network method to evaluate the effects of the two methods. As a more mature method of artificial intelligence, BP neural network is widely used in a wide range of applications and has the characteristics of strong generalization ability and fast convergence, so we choose it as the base model. The specific work of this paper is as follows: (1) in-depth study of the relevant theory of BP neural network (BPNN), focusing on the structure of BPNN and the working principle of algorithm; the problems to be solved in the clinical anesthesia effect evaluation have laid a theoretical foundation for the establishment of an improved BPNN evaluation model in the following chapters. (2) introduce the basic principle of genetic neural network, analyze the benefits of combining genetic neural network and BPNN; introduce in detail the process of genetic algorithm to optimize the weights and thresholds of BPNN, and establish a GA-BP evaluation model. The test proves the feasibility and superiority of the model.

## 1. Introduction

With the increasing number of major clinical operations and the need for severe treatment, arterial puncture and catheterization have become one of the main invasive monitoring techniques [1]. From the first case of radial artery puncture performed by humans, until today, such operations have been brilliant in operating rooms, ICUs, and interventional operating rooms. Arterial puncture and catheterization have a history of more than 300 years [2]. The main function of arterial puncture cannula is to monitor arterial blood pressure continuously in real time [3]. At the same time, it has many advantages. On the one hand, it can observe the fluctuation of blood pressure under special circumstances. On the other hand, the patient's volume status is assessed based on the arterial waveform, and fluid therapy is guided [4]. Despite the above-mentioned advantages, various factors can lead to failure of radial artery puncture and catheterization, and even complications. Some studies have summarized a series of complications related to arterial puncture and catheterization. The order of incidence is arterial spasm and occlusion, hematoma, infection, puncture site oozing, bacteremia, permanent ischemic injury, pseudoaneurysm, etc., the most serious complication is the ischemic injury of the puncture hand [5–7]. Clinical anesthesiologists are the main performers. When they have a certain working years and experience, the success rate of puncture and cannulation is not very different. The success rate of arterial puncture cannulation for beginners in anesthesia is generally low, and a long learning curve and a certain number of puncture cases are required to achieve a certain level of operation. The study found that the traditional puncture and tube placement method completely rely on the anesthesiologist's touch positioning and clinical experience, which has extremely high requirements for the anesthesiologist's operating skills and clinical experience. Due to the lack of operation experience for beginners, the failure rate is high, and it is easy to cause complications in patients [8]. With the improvement of modern ultrasound technology, arterial catheter ultrasound technology has been continuously applied. The application of ultrasound-guided arterial puncture and catheterization in clinical anesthesia has made its success rate higher and higher. Analysis of the application effect of ultrasound-guided arterial puncture and catheterization in clinical anesthesia plays an important role in the promotion of arterial catheterization ultrasound technology.

BP neural network is a multilayer feedforward network based on BP algorithm, whose network structure is simple, mature algorithm, has the advantages of self-learning and self-adaptation, and has the characteristics of nonlinear dynamics. BP algorithm trains the network through input and output data sample sets, according to the principle of error backward transmission, and its learning process includes the forward propagation process of information and the backward propagation of error, which are two processes for it is trained repeatedly, and the changes of network weights and deviations are calculated continuously in the direction of gradient descent of the relative error function, gradually approaching the target. Neural networks with their unique properties provide a completely new avenue for the study of machine learning. At present, neural networks have been applied to many aspects, such as pattern recognition, prediction, control of dynamic systems, and language learning. It is believed that in the future research and development, BP neural networks will be applied more widely, and more achievements will be made.

In the past ten years, the application of deep learning technology in the evaluation of medical effects has shown an increasing trend, and classification algorithms have been widely used in the study of treatment effects of various diseases [9, 10]. Reference [11] introduced the application of machine learning in medical images, mainly including the use of machine learning techniques to solve practical problems in “image recognition of lung cancer pathological cells” and “prostate CT image segmentation”. Reference [12] proposed a method combining transfer learning and convolutional neural network, which has a good effect in cancer image recognition. Reference [13] proposed a support vector machine-based pancreatic cancer detection method and found 12 characteristic genes closely related to pancreatic cancer. Reference [14] used semi-supervised learning of graph convolutional networks to predict whether a patient had cancer. Reference [15] proposed two improved support vector machine methods, SVM-PCA and SVM-RFE, for the diagnosis of cervical cancer and the evaluation of treatment effects. Based on the above research background, this paper uses neural network technology to evaluate the application effect of ultrasound-guided arterial puncture in clinical anesthesia. The main contributions of this paper are as follows: This study expounds the defects of the standard BP network and arterial puncture under ultrasound-guided needs to solve the problems in the clinical anesthesia effect assessment and build the improved BP network model for subsequent chapters that laid a theoretical foundation. This paper improves the traditional BP algorithm and uses the improved algorithm to find the appropriate number of hidden nodes in BP network. Second, according to the defects of BP network and the artery of ultrasound-guided puncture, the characteristics of the evaluation of clinical anesthesia, GA-BP evaluation model is established. Genetic neural network and BP network are analyzed in this paper, with the advantage of combination of introduced genetic algorithm to optimize the process of BP network weights and threshold, and through the test instance proves the feasibility and superiority of the model.

## 2. Related Work

As a “new stethoscope” for modern diagnosis and treatment, ultrasound plays an increasingly important role in the monitoring and management of patients in the fields of anesthesia, critical care, and emergency. In recent years, in clinical anesthesia work, with the continuous development and popularization of technology, ultrasound covers more and more fields, including airway ultrasound, gastric contents ultrasound, chest ultrasound, abdominal ultrasound, circulatory assessment, regional anesthesia, perioperative cardiac ultrasound, and ultrasound-guided vascular puncture, etc. [16–20]. Ultrasound will be a very important daily technique in clinical anesthesia practice. In recent decades, the range of ultrasound applications has continued to expand as the concept of whole-body point-of-care ultrasound has begun to be introduced into the anesthesiologist's technical field. Arterial puncture is usually used for critically ill patients or patients who are planning to undergo major surgery. Through the invasive arterial catheter, the patient's blood pressure can be monitored and continuously recorded in real time, which is convenient for clinicians to adjust the dose of vasoactive drugs in time, so as to maintain the patient's hemodynamics of stability. When patients require frequent arterial blood gas analysis, arterial blood can be obtained easily and conveniently through an arterial catheter. In addition, the arterial catheter can also be used as a means of interventional therapy such as cardiovascular. Arterial cannulation is one of the commonly used clinical techniques in anesthesia, emergency, and intensive care units [21–24]. Arterial cannulation is an essential skill for anesthesiologists. However, even experienced operators may encounter challenges when encountering neonatal patients, obese patients, shock, edema, arterial spasm, etc. Local hematoma at the puncture site or even failed puncture [25]. Although arterial catheterization is generally a relatively safe procedure, complications related to catheterization, including mechanical injury, infection, and thrombosis, still occur in 1% to 5% of patients. Because of its superficial location and the supply of blood to the hand together with the ulnar artery, the radial artery is the site of arterial puncture with the lowest complication rate, so it is the first choice for arterial puncture and catheterization [26]. Real-time ultrasound guidance can improve diagnostic and procedural accuracy, reduce patient anxiety and discomfort, reduce procedural-related complications, and spend less time with higher success rates. There are no absolute contraindications to ultrasound guidance. However, it should be noted that if the skin or soft tissue at the planned puncture site has infection or severe peripheral vascular disease, or abnormal blood supply to local tissues or organs, or the patient has severe coagulation system disease, the arterial puncture and catheterization itself is contraindicated [27–29]. In clinical practice, in many hospitals, ultrasound guidance has been routinely used for central venous catheterization, and many studies have demonstrated that ultrasound guidance can improve the first-time success rate and reduce complications [30]. In recent years, more and more studies have shown that ultrasound guidance can also improve the first-time success rate and reduce complications when it is used for radial artery puncture [31]. However, unlike the central vein, the diameter of the radial artery is small, and despite the use of ultrasound, its first-time success rate has not yet reached a satisfactory level. Therefore, in recent years, researchers have been trying to improve the ultrasound-guided radial artery puncture technique in order to improve the first-time success rate [32]. In clinical practice, with the rapid development and popularization of ultrasound technology, more and more operators will choose ultrasound salvage when they encounter difficulties in radial artery puncture, and even choose ultrasound guidance for the first operation. Unfortunately, there is currently no standard protocol for ultrasound-guided radial artery catheterization. However, ultrasound guidance has generally been recognized as an effective adjunct to arterial cannulation. Increasingly, ultrasound guidance is being employed in operating rooms, emergency departments, and critical care units at many medical facilities due to the advancement of ultrasound technology.

In recent years, efforts have been made to explore more reasonable evaluation methods at home and abroad, among which the artificial neural network evaluation method is widely used. Artificial neural network simulates the way of human thinking. It does not need to establish a certain model in advance for the judgment and classification of things and only adopts intuitive reasoning and judgment based on the essential characteristics of things [33]. Therefore, using artificial neural network to evaluate the application effect of ultrasound-guided arterial puncture and catheterization in clinical anesthesia will not be constrained by a certain model, making the evaluation results more objective. At present, the artificial neural network used for evaluation is mostly BPNN, namely error back propagation network and Hopfield network. For example, the literature [34] applied artificial neural network to the effect evaluation of arterial puncture and catheterization in clinical anesthesia. The results show that artificial neural network has strong adaptability in this type of evaluation, and the evaluation results are objective and reasonable. As a result, this paper provides an overview of the BP neural network's structure and algorithmic workings, as well as an analysis of the network's major flaws. It also summarizes the challenges associated with applying the BPNN to the evaluation of arterial puncture and cannulation, and it offers a method for doing so. The establishment of the evaluation model for arterial puncture and catheterization based on the improved BPNN has laid a theoretical foundation.

## 3. Method

### 3.1. Introduction of BP Neural Network

BPNN has three layers: an input layer, a hidden layer, and an output layer. There is one input layer and one output layer, as well as the possibility of many hidden levels [16–18]. Each layer is connected by multiple neuron nodes, although nodes within the same layer are connected. Due to the lack of coupling between nodes in the same layer, neurons in each layer are only responsive to the input of neurons in the preceding layer; the output of neurons in each layer has no effect on the output of the preceding layer. BPNN's structure is seen in Figure 1.

(1) Input layer: depending on the situation, the number of processing units may be utilized to indicate the number of network inputs [19]. Use a linear transfer function, that is, *f*(*x*) = *x*.
(2) Hidden layer: used to represent the interaction between input processing units and all use nonlinear transformation functions. The number of processing units is determined by network debugging or empirical formula:
  (1) $$\begin{array}{c} H=\frac{\left(a+b\right)}{2}, \end{array}$$
where *H* is the number of hidden layer nodes, *a* is the number of input nodes, and *b* is the number of output nodes.
(3) Output layer: used to represent the number of outputs of the network. The number of processing units depends on the actual problem, and a nonlinear conversion function is used [20]. The most commonly used nonlinear transfer function is the hyperbolic function:
  (2) $$\begin{array}{c} f\left(x\right)=\frac{1}{1+e^{x}}. \end{array}$$

In the formula, when the independent variable *x* tends to positive or negative infinity, the function value tends to be constant, and its value range is [0, 1].

The input data of the network *I*=(*I*_1_, *I*_2_,…, *I*_*n*_) first pass through the hidden layer nodes from the input layer, and then reach the output layer node, and finally obtain the output data *O*=(*O*_1_, *O*_2_,…, *O*_*m*_). A neural network can be viewed as a highly nonlinear mapping from input to output:

(3) $$\begin{array}{c} f\left(I\right)=O. \end{array}$$

In practical applications, a BPNN with multiple hidden layers may be used. There is no accurate and effective theory and method for how to reasonably select the number of hidden layers and the number of nodes in the hidden layer of the BP network. The number of nodes in the input layer of the BP network is determined by the dimension *n* of the input vector *I*=(*I*_1_, *I*_2_,…, *I*_*n*_) of the training sample, and the number of nodes in the output layer is determined by the dimension *m* of output vector *O*=(*O*_1_, *O*_2_,…, *O*_*m*_).

If a three-layer BP neural network can be used to estimate any continuous function in a closed interval, it can also complete any mapping from n-dimensional space to three-dimensional space [21]. Even if two hidden layers are more likely to fall into local minima than one hidden layer, the BP network with two hidden layers is more difficult to train.

### 3.2. Improved Algorithm of BP Algorithm

Although BPNN is one of the most widely used neural networks, it has many significant advantages, but it also has its shortcomings, mainly in the following three aspects. (1) The BPNN has a slow convergence rate. (2) It is easy to fall into a local minimum, and the network training is more likely to fail. (3) The number of hidden layer nodes is difficult to determine. It is precisely because of the defects of the BP network that it encounters some difficult problems in the application process, which greatly limits the further development and application of the BP network. As a result, this work employs the novel GA-BP method to build the evaluation model, which is created by merging the genetic algorithm with the BP algorithm. The genetic algorithm is capable of doing both macroscopic and global optimization. Another advantage of this approach of searching is that it does not depend on higher order information like gradients, and it may be utilized in a distributed fashion for complicated non-linear problems that are difficult to solve with standard search methods. BPNN weights and thresholds may be optimized using a genetic algorithm with BPNN. The traditional BP neural network agent model has the problems of insufficient fitting accuracy and low computational efficiency. The GA-BP neural network agent model is established by optimizing the initial weights and thresholds of the BP neural network using genetic algorithm (GA). The GA-BP neural network was trained to further improve the accuracy of the GA-BP neural network agent model. Although the above research has improved the fitting accuracy and computational efficiency of the agent model to a certain extent, the BP neural network model established based on GA still has problems such as premature maturation and slow convergence, and its optimization effect has certain limitations. Based on this, this paper introduces the thinking evolutionary algorithm (MEA) to optimize the initial weights and thresholds of the BP neural network, uses the BR algorithm to train the network that obtains the optimal initial values, proposes a reliability calculation method based on the MEA-BR-BP neural network agent model, and takes a truck bogie frame as an example to calculate its reliability, so as to verify the superiority of the method proposed in this paper. The following are the particular measures to take.

(1) Coding and the process of creating the first round of inhabitants: The real number coding technique was used since the network weight is a real number. A real number array is formed by cascading the BPNN's weights and thresholds in the correct sequence to construct a genetic algorithm's “chromosome.” A three-layer BP network topology is used in this article, and the number of nodes in the input layer, hidden layer, and output layer is set to be *n*_1_, *n*_2_, and *n*_3_, respectively, then the length of the encoding is
  (4) $$\begin{array}{c} L=n_{1}\times n_{2}+n_{2}\times n_{3}+n_{2}+n_{3}. \end{array}$$
 Randomly generate *m* chromosomes of length *L*, that is, to form an initial population. For the determination of the population number *m*, if it is too large, the network will converge slowly; if it is too small, it will reduce the network training accuracy.
(2) Determination of fitness function: assign the *L* connection weights in the initialized population to the BPNN, carry out the forward propagation of the input signal, and calculate the sum of squared errors *E*(*i*) between the output value of the network and the expected output. Set the given fitness function as follows:
  (5) $$\begin{array}{c} f\left(i\right)=\frac{1}{E\left(i\right)}. \end{array}$$
 In this way, the evaluation criteria of genetic algorithm and BP network can be integrated. Therefore, the higher the fitness f(k), the better the network performance.
(3) Fitness sorting: choose the proportional method for selection, that is, first calculate the fitness of each individual in the population, and then sort all the individuals in the group according to their fitness, so as to assign the probability of each individual which is selected.
  (6) $$\begin{array}{c} P_{L}=\frac{f\left(i\right)}{\sum_{i=1}^{L}f\left(i\right)}. \end{array}$$
 It can be seen from formula (6) that the individual with higher fitness is more likely to be selected, and the individual with lower fitness is less likely to be selected.
(4) Generation of new population: To create new populations, employ crossover and mutation operators to operate original people, insert new individuals into the original population, and establish new populations. It is determined whether or not the new population's fitness passes the optimization requirement by calculating its connection weight and comparing it to the BPNN.
(5) Generation of initial weights of BP network: Individuals are decoded after achieving a defined performance index or a maximum genetic algebra to get the ideal network connection weight coefficient. Thereafter, the method terminates when error squared sums equal or exceed the required accuracy or the stated maximum number of iterations, depending on how many iterations it takes to train the network.

### 3.3. Determination of Network Topology

Whether the determination of the network structure is reasonable directly affects the objectivity and accuracy of the evaluation results and the applicability of the network model. BP artificial neural network model establishment relies in large part on the derivation of topological structure. Number of layers, nodes and layers, as well as the number of hidden layer levels, and the number of hidden layer nodes are all factors in determining network structure. 1) The number of network layers: the number of hidden layers determines the number of network levels in the BPNN architecture since the input and output layers are required. The performance of the network is closely related to the number of hidden layers selected. 2) An input layer, a hidden layer, and an output layer make up the three layers of the network model described in this research. Node count in the input and output layers: Table 1 shows the results of our examination of eight evaluation indicators:

Therefore, it can be determined that the number of nodes in the input layer is 8. There is 1 output node, and the final output result is determined according to the total score of all 8 indicators. According to the score, it is divided into 5 levels: 1, 2, 3, 4, and 5. Level 1 represents the best effect, and level 5 represents the worst effect. 3) Determination of the number of hidden layer nodes: according to the following formula, the range of hidden layer nodes is determined as [4, 13]

(7) $$\begin{array}{c} h=\sqrt{n+m}+a,\;a\in \left[1,10\right]. \end{array}$$

Finally, the number of hidden layer nodes when the best effect is obtained through experiments is 8.

### 3.4. Determination of Experimental Group and Control Group

Arterial puncture is a common invasive procedure that can monitor blood pressure in real time, assess volume responsiveness, and provide convenient access for blood gas monitoring. Radial, cubital, and femoral arteries can be used as puncture points. To puncture these blood vessels, most doctors choose to utilize the superficial radial artery because to its minimal risk of problems, its dual blood supply to and from the hand (radial and ulnar arteries), and its location on the hand. In order to better highlight the application effect of ultrasound-guided arterial puncture in clinical anesthesia, a control group and an observation group were selected in this paper. Patients in the control group received the traditional touch positioning method. The anesthesiologist's left hand needs to explore the position of the patient's radial artery pulsation in a horizontal direction. He holds the needle in his right hand and inserts the needle at an angle of 30 degrees. The observation group underwent ultrasound-guided arterial puncture. The anesthesiologist holds the ultrasound probe in his left hand and checks the patient's arterial position and needle insertion point with his left hand. He holds the needle in his right hand and injects the needle at a 30-degree angle. Ultrasound showed effort to enter the inside of the radial artery, and when the blood returned, the needle was reinserted 1 to 2 mm.

## 4. Experiment and Analysis

### 4.1. Data Set

To test whether a network model can reflect the laws contained in the sample, that is, whether it has the ability to generalize, it must be evaluated by the size of the nontraining sample error. Therefore, this paper divides the total samples into two parts: training samples and test samples and uses the mean square error of the test samples to judge the quality of the network. In this paper, Matlab is used to build the network. The hidden layer neuron transfer function in the network adopts the sigmoid tangent function, the output layer neuron transfer function adopts the pure linear function purelin, and the training function adopts the trainlm, that is, the LM algorithm. The learning rate is set to 0.5, the expected error is 0.001, and the maximum number of times the network is trained is 1000. The samples in this paper are from a total of 1000 research subjects who have received traditional touch positioning method and ultrasound-guided positioning method in a tertiary hospital.

After the network is built, 200 groups are selected from the 1000 groups of samples as test samples, and the rest are used as training samples to train the network, and the cycle times of each network model and the mean square error of the training samples are recorded. Since the weight threshold of the neural network is different each time it starts training, even if the network with the same topology structure, the number of cycles for each training and the final mean square error are different. Respectively train multiple times and take the best one to obtain the data. The part of the sorted data set is shown in Table 2. The index in Table 2 is represented by each label in Table 1. The experimental environment of this article is as follows: the hardware environment is Linux system, NVIDIA GTX 3080; the software environment is Python3.7, sklearn0.20.2, and other toolkits. The proposed method in this paper of training data set on the 20 epochs (round). Training method is as follows: model of the initial vector is set to 0.0001; use the Adam optimizer; batch size is set to 8 (batch size refers to the choice of a training sample size and the size of device GPU limitation, according to the model to select the best optimization and speed).

### 4.2. Experiment to Determine the Number of Nodes in the Hidden Layer

According to the description in Chapter 3, the number of nodes in the hidden layer ranges from 4 to 13, so this paper selects the number of nodes as 4, 6, 8, 10, 12, and 14 to simulate, respectively. Finally, the number of hidden layer nodes with the best effect is determined according to the experimental results, see Figures 2–4 for details. In this paper, we use the mean squared error (MSE) as a loss function, which is common in machine learning. In mathematical statistics, the mean squared error is the expected value of the squared difference between the parameter estimate and the parameter value, which is called MSE. MSE is a convenient way to measure the “mean error”, which can evaluate the degree of variation of the data.

Comparing the experimental results in Figure 2-figure supplement 4, we can see that when the number of hidden nodes is 8, its convergence speed is the fastest, and it reaches convergence at the 10th epoch. Moreover, its performance at convergence is optimal and the training effect is the best, so the number of hidden layer nodes chosen in this paper is 8.

### 4.3. Comparison of the Experimental Results of the Two Methods

In order to ensure the rationality and authority of the set evaluation level, the chief physician of clinical anesthesia for arterial puncture was invited to set the evaluation level corresponding to the score reasonably. The final experimental results are shown in Table 3.

Based on the above experimental results, the observation group used ultrasound-guided arterial puncture and catheterization, the success rate was higher than that of the traditional touch positioning method, and the occurrence of adverse reactions of patients was also reduced. Therefore, ultrasound visualization technology will more effectively analyze the arterial blood situation and accurately determine the patient's puncture point and needle insertion direction. In addition, the anesthesiologist will also effectively analyze the specific location of the needle and artery during the puncture and catheterization and be combined with the actual situation to realize the adjustment of the puncture needle position and the puncture needle angle. In the case of promoting the success rate of puncture, it will also reduce the incidence of complications. Therefore, ultrasound-guided arterial puncture cannulation has higher advantages.

## 5. Conclusion

There is ample evidence that ultrasound-guided arterial puncture is superior to traditional palpation, both in terms of success rate and complications. The advantages of ultrasound guidance are not limited to arterial cannulation associated with surgical anesthesia. Recent studies have found significant advantages of ultrasound guidance when arterial blood gas extraction is difficult in other in-hospital locations outside the operating room. At present, most researches are devoted to improving the puncture technique to add the success rate and reduce the complication rate. Studies have shown that a superficial puncture site is more likely to penetrate the posterior wall or form a local hematoma. This is different from the traditional palpation method to puncture the artery. When using the palpation method, in order to facilitate the palpation of the pulse, it is usually selected at the superficial position of the distal end of the radial artery, and the increase of the depth that will increase the difficulty of puncturing. Unlike ultrasound guidance, it is not limited by depth. Finally, this paper completed the following work. Further study of the theory of BP neural network, BP network is the main research of the structure and working principle of the algorithm. Expounds the defects of standard BP network and arterial puncture under ultrasound-guided needs to solve the problems in the clinical anesthesia effect assessment, build the improved BP network model for subsequent chapters laid a theoretical foundation. In this paper, the traditional BP algorithm was improved, by using the improved BP network algorithm to find the suitable number of hidden layer nodes. Second, ga-BP evaluation model was established according to the defects of BP network and the characteristics of clinical anesthesia evaluation of ultrasound-guided arterial puncture. Genetic neural network and BP network are analyzed in this paper, with the advantage of combination of introduced genetic algorithm to optimize the process of BP network weights and threshold, and through the test instance proves the feasibility and superiority of the model. The experimental results demonstrate that the improved BP algorithm proposed in this paper can overcome the shortcomings of the BP algorithm, which tends to fall into local minima, and at the same time, the generalization ability of the neural network can be exploited to improve the application of ultrasound-guided arterial puncture cannulation in clinical anesthesia. In our future work, we plan to conduct a study on the application of overly convolutional neural networks to ultrasound-guided arterial puncture cannulation in clinical anesthesia.

## Figures and Tables

**Figure 1:** BP network structure diagram.

**Figure 2:** Training effect when *N* = 4 and *N* = 6.

**Figure 3:** Training effect when *N* = 8 and *N* = 10.

**Figure 4:** Training effect when *N* = 12 and *N* = 14.

**Table 1:** Evaluation indicators.

Index	Label	Score
One-time penetration success rate	X1	1–5
Failure rate	X2	1–5
Penetration catheter placement rate	X3	1–5
Total puncture catheter time	X4	1–5
Time to penetrate the target vessel	X5	1–5
Number of puncture points	X6	1–5
Adverse reaction ratio	X7	1–5
Number of times to change the needle direction	X8	1–5

**Table 2:** The part of the sorted data set.

NumIndex	1	2	3	4	5	6	7	8
X1	2	4	4	2	2	2	4	1
X2	3	5	4	3	3	3	4	2
X3	2	3	5	4	2	3	5	2
X4	4	4	5	3	4	3	2	4
X5	1	3	2	3	4	2	2	3
X6	2	4	3	2	4	4	3	3
X7	3	2	4	1	5	3	5	2
X8	1	5	5	4	4	2	4	4

**Table 3:** Comparison of experimental results between the two methods.

Num.	Ultrasound guided output	Traditional method output	Authoritative physician evaluation
1	4	4	4
2	5	5	5
3	4	4	4
4	5	4	5
5	4	3	4
6	4	3	4
7	3	4	3
8	2	1	2
9	5	5	5
10	4	3	4

## Data Availability

The data sets used during the current study are available from the corresponding author on reasonable request.
